The article "Multitarget Detection and Tracking Method in Remote Sensing Satellite Video" was published in 2021. Journal: Comput Intell Neurosci.

# Multitarget Detection and Tracking Method in Remote Sensing Satellite Video

**DOI:** 10.1155/2021/7381909

**Published:** 2021-08-31

**Authors:** Lei Lei, Dongen Guo

**Affiliations:** School of Computer and Software, Nanyang Institute of Technology, Nanyang 473000, China

## Abstract

A remote sensing video satellite multiple object detection and tracking method based on road masking, Gaussian mixture model (GMM), and data association is proposed. This method first extracts the road network from the remote sensing video based on deep learning. In the detection stage, the background subtraction algorithm is used based on the GMM to obtain the detection results of the moving targets on the road. In the tracking stage, the data association of the same target detection result in adjacent frames is realized based on the neighborhood search algorithm, so as to obtain the continuous tracking trajectory of each target. The experiments about multiobject detection and tracking are conducted on data measure by real remote sensing satellites, and the results verified the feasibility of the proposed method.

## 1. Introduction

At present, with the rapid development of aerospace technology and the gradual deepening of remote sensing applications, the demand for high-resolution satellite remote sensing applications has gradually shifted from static reconnaissance to real-time dynamic monitoring. A series of video satellites have been deployed in recent years. The video satellite can obtain the submeter resolution color dynamic video through the staring imaging mode and obtain continuous video image data of the area of interest, which is particularly suitable for regional dynamic change monitoring, such as situation changes, dynamic target reconnaissance and surveillance, and attack effect evaluation [1–4]. At the same time, it can also meet various civil needs such as antiterrorism, disaster prevention and relief, and intelligent traffic control. Therefore, improving the intelligent processing level of the remote sensing video satellite multiobject detection and tracking algorithm can greatly reduce the degree of manual participation in the information extraction process, which could bring important promotion significance to the development aerospace information industry and social and economic progress.

In this context, this paper focuses on video satellites, an emerging aerospace remote sensing technology, and performs fully automatic, high-precision, and high-speed information extraction of dynamic remote sensing videos acquired by video satellites in the “gaze” imaging mode. A target detection and tracking algorithm is developed for the videos measured by remote sensing satellites. In existing research, satellite video detection and tracking methods are mainly inherited from traditional video detection and tracking methods. In the detection process, the main methods can be divided into frame difference method, optical flow method, and background subtraction method. The frame difference methods perform dynamic target detection by judging the difference between the two frames before and after [5, 6]. The optical flow methods collect the instantaneous changing rate of the gray levels when the object is moving in the optical flow field. Those changes can reflect the change of the image, so the moving target can be inspected by the optical flow [7, 8]. The background subtraction methods first establish a background model to represent the scene and then compare the following frames with the model. By properly performing the subtraction, the result is assumed to be the movement area [9, 10]. In the tracking process, the main methods can be divided into traditional filtering, correlation filtering, and deep learning ones. Traditional filtering methods mainly include mean shift algorithm, Kalman filter algorithm, and particle filter algorithm [11, 12]. The correlation filter tracking algorithm essentially trains the filter according to the first frame of the target sample, which is used to search for the area where the target is located, and judges the target position according to the response value. Then, the filter is constantly updated during the tracking process [13, 14]. The tracking algorithms based on deep learning are mainly divided into two categories [15, 16]: one is to design tracking algorithms based on deep features and related filtering; the other is to track targets' end-to-end based on deep networks. The existing satellite video target detection and tracking algorithms basically follow the related results in traditional video processing, as shown in [17–27]. Aiming at the needs of satellite video moving target detection and tracking, this paper proposes a background subtraction method based on a hybrid Gaussian background model combined with a road mask. The proposed method can significantly reduce the missing detection of target pixels due to the changes in illumination and shadows. In the experiment, the performance of the proposed method is tested based on real satellite video data, and the results verify its effectiveness.

The article "Multitarget Detection and Tracking Method in Remote Sensing Satellite Video" was published in 2021. Journal: Comput Intell Neurosci.

## 2. Preprocessing of Remote Sensing Satellite Video

The preprocessing of remote sensing video data can realize automatic enhancement processing of high-resolution remote sensing video images, including video processing functions such as color enhancement, edge enhancement, and noise removal. The preprocessing could improve the visual effect and interpretability of remote sensing video. The video quality and amount of information can be enriched to strengthen the effect of video discrimination and recognition, thus providing data support for subsequent information extraction. At the same time, the preprocessing operations also include the orthorectification of the remote sensing image. After the remote sensing image is orthorectified, one of the important tasks is to accurately match the remote sensing image with the geographic coordinates so that the remote sensing image coordinates and geographic information are linked, so as to facilitate the extraction of useful information. Aiming at the geometric distortion of remote sensing images caused by the imaging system and terrain and other factors, a remote sensing image orthorectification technology based on rational polynomial coefficient (RPC) parameters is realized. By analyzing the RPC information in the image metadata and importing the digital elevation model (DEM), the conversion relationship between the image row and column number coordinates and the WGS84 latitude and longitude coordinates is obtained. The projection transformation is performed according to the conversion relationship using the image reprojection method to realize the remote sensing image ortho correction processing. After orthorectification, the remote sensing image can have both the characteristics of the topographical map and image. It has high accuracy and rich information in areas with large terrain undulations.

## 3. Methodology for Detection and Tracking

### 3.1. Target Detection

Considering the application requirements of high-resolution satellite imagery for detection and recognition of interested targets, the popular deep learning algorithm is introduced into the remote sensing application field. For remote sensing image target recognition and detection, a typical algorithm based on deep learning is developed. By constructing a database of typical remote sensing targets, the automatic identification and detection of targets such as aircraft, ships, airports, and ports can be realized. For the same type of target, for different application scenarios, a fast model and a high-precision model are constructed through algorithm tuning. Based on the rich texture information of high-resolution satellite images, a deep convolutional neural network structure and target detection algorithm framework are constructed, and multilayer feature extraction and multifeature fusion are performed on high-resolution optical satellite images to improve the accuracy of target recognition. The improved faster R-CNN and Resnet algorithm [28–31] are used to train the training dataset to realize the intelligent target detection of high-resolution remote sensing images and realize the high-precision intelligent target detection technology for high-resolution satellite images. After the object detection is completed, the number of objects and the latitude and longitude information can be output. The main process of the target detection and recognition algorithm for a specific target is described as follows:

  Step 1: the ImageNet model is used to initialize and independently train a Region Proposal Network (RPN).
  Step 2: the proposal generated by the RPN network in Step 1 is used as the input to initialize the ImageNet model and train a Fast R-CNN network. The parameters of each layer of the two networks are not shared.
  Step 3: the Fast R-CNN network in Step 2 is used to initialize a new RPN network. The learning rate of the RPN and Fast R-CNN is set to 0. Only the network layer unique to RPN is updated. After retraining, the two networks share all common convolutional layers.
  Step 4: the shared network layer is fixed, and it combines with the fast R-CNN unique network layer to form a unified network, which continues training and completes the fine-tuning of the fast R-CNN unique network layer.
  Step 5: based on the trained target detection and recognition model parameters, automatic target detection is performed on objects of interest (such as airplanes, oil tanks, and buildings) and other objects of interest.

The article "Multitarget Detection and Tracking Method in Remote Sensing Satellite Video" was published in 2021. Journal: Comput Intell Neurosci.

### 3.2. Detection and Tracking of Moving Targets

Aiming at the characteristics of continuous video images obtained by video satellites for gaze observation of a certain area, high-resolution satellite video dynamic vehicle detection and tracking are realized. The algorithm first uses the background subtraction method based on the road mask processing and the Gaussian mixture model (GMM) to initially extract the moving vehicles. At the same time, it uses the geometric characteristics of the vehicle to filter the preliminary extraction results and employs the quadratic curve fitting method based on the least squares method to track the moving vehicles.  Figure 1 shows the detection and tracking process of dynamic targets on the road. The specific steps can be described as follows:

First, extract the stabilized video frames in sequence, and preprocess the video frame images to strengthen the image discrimination and recognition effect. For the satellite video, use the Gaussian mixture background modeling method based on the statistical information of pixel samples to estimate the background, use the statistical information such as the probability density of a large number of sample values of the pixels in a long time to represent the background, and then, use the statistical difference to determine the target pixel and model complex dynamic backgrounds. In the Gaussian mixture background model, it is considered that the color information between pixels is not related to each other, and the processing of each pixel is independent of each other. For each pixel in the video image, the change of its value in the sequence image can be regarded as a random process of continuously generating pixel values, that is, the Gaussian distribution is used to describe the color of each pixel and the regularity of single-mode and multi-mode state. For the multimodal Gaussian distribution model, each pixel of the image is modeled by the superposition of multiple Gaussian distributions with different weights. Each Gaussian distribution corresponds to a state that may produce the color of the pixel, and the weight of each Gaussian distribution and the distribution parameters are updated over time.

The article "Multitarget Detection and Tracking Method in Remote Sensing Satellite Video" was published in 2021. Journal: Comput Intell Neurosci.

Then, the moving target in the satellite video is detected. Using the background difference method, mathematical morphology and statistical analysis of the obtained connected domains are performed, and a global threshold is calculated to binarize the image. Background subtraction first establishes a background model to represent the scene, then compares the following frames with the model and performs subtraction, and the result is the motion area. When using background subtraction to detect moving targets, the difference between the model of the background image and the real scene will affect the target detection performance. Therefore, by judging the area of the connected region of the moving targets, the noise can be filtered out to increase the detection accuracy.

Finally, the extracted moving target is tracked. By counting the centroid position, pixel area, and average gray information of each moving target in the foreground, the target tracking decision is established considering the deformation and gray value changes of the same target in different frames due to illumination, occlusion, etc. The following figure shows the flowchart of the moving target tracking algorithm. When tracking the target, use the quadratic curve fitting method based on the least squares method to predict the vehicle position in the next frame according to the obtained data of the target, obtain the predicted centroid position, and search in the neighborhood of the predicted centroid position. Matching can greatly increase the search speed and reduce the calculation complexity and calculation time. After tracking the moving target frame by frame, according to the relative position of the front and rear frames, the solution of the motion parameters of the moving target including the motion direction and the motion speed can be realized.

The article "Multitarget Detection and Tracking Method in Remote Sensing Satellite Video" was published in 2021. Journal: Comput Intell Neurosci.

#### 3.2.1. Extraction of Road Mask

Generally, the dynamic target is located on the roads in the remote sensing image. Therefore, in order to further reduce the number of false alarms and calculation load, the road network extraction algorithm used in this paper combines deep learning and high-resolution satellite image data [28–31]. This method can automatically and accurately extract the road network information of the area that cannot be obtained by traditional surveying and mapping methods. Based on deep learning technology, it can quickly and accurately realize the pixel-level classification of remote sensing images and learn high-level abstract features through deep convolutional neural networks to improve classification accuracy. For classification results, the classification postprocessing functions are designed, including classification merging and classification information statistics.  Figure 2 shows an example of road mask extraction. Comparing the original image and the extracted road mask, it can be seen intuitively that this method can realize the extraction of highways with good precision. Most of forest roads, rural roads, and other small roads can be effectively separated from the surrounding buildings, trees, etc.

#### 3.2.2. Video Registration

The scale invariant feature transformation (SIFT) features and GPU acceleration technology are used to achieve subpixel level registration. The SIFT feature is an image local feature description operator that is based on scale space and maintains invariance to image scaling, rotation, and even affine transformation. This feature has the characteristics of uniqueness, versatility, and scalability. It is used in the field of image registration with wide range of applications. The traditional SIFT feature matching algorithm is slow and has poor applicability to ultrahigh resolution remote sensing images. The GPU acceleration technology is used to achieve rapid extraction and matching of feature points of ultralarge resolution remote sensing images.

#### 3.2.3. Background Difference

There are *K* Gaussian models used to characterize each pixel feature in a single frame of the video satellite image, which updates the GMM after a new frame of image is obtained. And, each pixel in the current image is used to match the GMM. If it succeeds, it is determined that the point is a background point. Otherwise, it is the former scenic spot. A square structure with the size of 3 × 3 is used for the closing operation (expansion before corrosion). The area of connected domains (8 neighborhoods) is counted in the foreground to remove the connected domains whose area is less than or greater than a certain threshold range.

The article "Multitarget Detection and Tracking Method in Remote Sensing Satellite Video" was published in 2021. Journal: Comput Intell Neurosci.

#### 3.2.4. Multiobject Detection and Tracking Algorithm

A two-dimensional index table is created to record the position of the target in a single frame and search in the neighborhood of the predicted centroid. The predicted centroid is the position information of the centroid of the vehicle to be confirmed or obtained from the previous frames. Then, the quadratic function fitting is performed to obtain the predicted position of the current frame. There are several indexes to evaluate the tracking performance. The first is the number of missing targets. When there is no hypothetical position of the target in the current frame, the prediction area of the target in the current frame is not found. The second is the number of misjudgments. The given position assumes that there is no tracking target corresponding to it. The third is the number of mismatches. This problem mostly occurs in the case of occlusion or adhesion caused by multiple target positions too close.

## 4. Experiments and Analysis

This paper uses a piece of real remote sensing video for target detection and tracking to test the performance of the proposed method. The experiment runs on the Matlab platform, and the hardware requirement is Core i7-3770 CPU (memory 3.4 GB).

### 4.1. Detection of Moving Targets

Figure 3(a) shows a video satellite shot of a city road scene. It can be seen that there are dense dynamic vehicle targets on the road. The size of the vehicle target is limited, and it is usually embodied as an extended point target on the image. Due to the small size of the vehicle target, it is difficult to use the detection network based on deep learning to obtain the detection results. The proposed method first uses the road mask to remove the building areas on both sides of the road, so as to avoid the false alarms outside the road area. Afterwards, for the targets on the road, the interframe difference method based on GMM is used to obtain the detection result of the dynamic target, as shown in Figure 3(b). Compared with the original image, it can be found that the detection result reflects the vehicle target in the image well, which provides a good foundation for subsequent target tracking.

### 4.2. Target Tracking

In this paper, a data association algorithm based on nearest neighbor search is used to correlate the dynamic target detection results of two adjacent frames to obtain the continuous tracking trajectory of the dynamic target. As shown in Figure 4, Figures 4(a) and 4(b) are adjacent frames in the remote sensing video. Compared with Figure 4(a), the vehicle target in Figure 4(b) has a slight displacement, which is much smaller than the geometric distance between different moving targets. Therefore, by performing the nearest neighbor search with a radius around the detection result of each dynamic target in Figure 4(a), the corresponding detection result of the target in Figure 4(b) can be obtained. By associating two corresponding detection results, the proposed method can obtain the tracking results of the dynamic target between two adjacent frames.

The article "Multitarget Detection and Tracking Method in Remote Sensing Satellite Video" was published in 2021. Journal: Comput Intell Neurosci.

In order to quantitatively evaluate the performance of the proposed method, the Intersection over Union (IoU) index is calculated [30, 31]. Given the bounding rectangle for detection and tracking of each target and the artificially labeled truth rectangle, the IoU value is defined as follows:

(1) $$\begin{array}{c} \text{IoU}=\frac{\left|r_{t}\cap r_{g}\right|}{\left|r_{t}\cup r_{g}\right|}, \end{array}$$

where ∩ and ∪ represent the intersection and union of two regions and |·| represents the number of pixels in the region. In order to measure the performance of the detection and tracking algorithm on a certain video, the number of frames whose IoU value is greater than a given threshold is counted.

Figure 5 shows the corresponding IoU values for different search radii. It can be seen that when the search radius is 4 pixels, the detection and tracking algorithm proposed in this paper can reach 92.8%, and almost all targets can be detected and tracked correctly. The experimental results verify the effectiveness of the proposed method.

## 5. Conclusion

With the development of remote sensing technology, the spatial resolution, temporal resolution, and spectral resolution of future video satellites will become much higher. Also, the measured satellite video will become much clearer so the information that can be obtained through the video will also increase significantly. The dynamic target detection and tracking method of the video satellite remote sensing video data studied in this paper can improve the remote sensing satellite's reconnaissance capability of the dynamic mobile small target. It can be seen from the experimental results that the proposed method successfully extracts the road mask information from the satellite video and uses GMM and background subtraction to extract the detection results of moving targets. The continuous motion of each target between different frames can be found using data association to realize the detection and tracking of the target of interest.

## Figures and Tables

**Figure 1:** Procedure of detection and tracking of moving targets.

The article "Multitarget Detection and Tracking Method in Remote Sensing Satellite Video" was published in 2021. Journal: Comput Intell Neurosci.

**Figure 2:** Illustration of road mask extraction in remote sensing images. (a) Original image. (b) Extracted road mask.

**Figure 3:** Illustration of moving targets detection in the remote sensing video. (a) Remote sensing image. (b) Detection results of moving targets.

**Figure 4:** The target detection results in two neighboring frames. (a) Former frame. (b) Latter frame.

**Figure 5:** The IoU values at different searching radius.

## Data Availability

The data used to support the findings of the study are available from the corresponding author upon request.
